The article "Relationship between miR-338-3p and Clinicopathological Parameters, Prognosis, and STAT3 mRNA Expression in Nasopharyngeal Carcinoma" was retracted in 2023. Reasons: unreliable results or conclusions; concerns about the data; concerns about the peer review; concerns about the citations.

# Relationship between miR-338-3p and Clinicopathological Parameters, Prognosis, and STAT3 mRNA Expression in Nasopharyngeal Carcinoma

**DOI:** 10.1155/2021/2681683

**Published:** 2021-10-19

**Authors:** Youyou Wang, Huijun Ren, Zhaohu Pan, Ben Liu, Fan Lin

**Affiliations:** Department of Otorhinolaryngology, Taizhou Hospital of Zhejiang Province Affiliated to Wenzhou Medical University, Taizhou, Zhejiang 317000, China

## Abstract

**Objective:**

To investigate the expression of miR-338-3p in nasopharyngeal carcinoma (NPC) and its relationship with STAT3 mRNA expression as well as their relationship with clinical pathological parameters and prognosis of patients.

**Methods:**

From September 2016 to September 2018, 71 patients with NPC were selected as the NPC group, and 71 samples of NPC tissues were collected during the operation. A total of 23 patients who underwent biopsy due to chronic nasopharyngitis were selected as the control group and 23 nasopharyngeal mucosal tissues were collected. The expressions of miR-338-3p and STAT3 mRNA in nasopharyngeal tissue of two groups were detected by real-time quantitative PCR, and the relationship between the two was analyzed. To collect clinical data of NPC patients and analyze the relationship between the expressions of miR-338-3p and STAT3 in NPC tissues and clinical pathological parameters of the patients, we followed up the patients with nasopharyngeal carcinoma for three years to observe the relationship between miR-338-3p, STAT3, and the prognosis of the patients.

**Results:**

The relative expression levels of miR-338-3p in nasopharyngeal tissues of the NPC group and the control group were 0.39 ± 0.05 and 1.01 ± 0.09, respectively (*P* < 0.05). The relative expression levels of STAT3 mRNA in nasopharyngeal tissues of the NPC group and the control group were 3.82 ± 0.21 and 1.04 ± 0.11, respectively (*P* > 0.05). miR-338-3p was negatively correlated with the relative expression of STAT3 mRNA in nasopharyngeal carcinoma (*r* = 0.038, *P* > 0.05). The expression of miR-338-3p was related to the age of the patient, clinical TNM stage, T stage, and distant metastasis (all *P* < 0.05). STAT3 expression was correlated with clinical TNM stage, T stage, and distant metastasis in our patient (*P* < 0.05). The expressions of miR-338-3p and STAT3 in nasopharyngeal carcinoma tissues from different gender, histological type, N stage, M stage, and degree of differentiation showed no statistical differences (*P* > 0.05). The survival rate of the group with low miR-338-3p expression was significantly lower than that of the group with high miR-338-3p expression (*P* > 0.05). The survival rate of patients with the high STAT3 expression group was significantly lower than that of patients with the low STAT3 expression group (*P* > 0.05).

**Conclusion:**

There is a negative correlation between the low expression of miR-338-3p and the high expression of STAT3 in NPC, which are all related to the TNM stage, T stage, and prognosis of the patient.

## 1. Introduction

The main reason why malignant tumors are difficult to cure is that they are not easy to be found in the early stage. Once obvious symptoms appear, most of them have reached the middle and advanced stage and formed a wider infiltration or metastasis, resulting in poor clinical treatment effect. It is generally believed that valuable biomarkers can significantly improve the survival rate by early diagnosis, assessment of prognosis, and guidance of treatment of the disease [1]. At present, the best antitumor therapeutic strategy still depends on early detection and close monitoring of early recurrence so that the therapeutic regimen can be reasonably adjusted. Finding molecular markers and early diagnostic methods for early diagnosis of tumors has always been the key to tumor prevention and treatment research. Nasopharyngeal carcinoma (NPC) is one of the common malignant tumors in the head and neck, and its incidence rate is about 50% of the primary malignant tumors of epithelial origin in the head and neck. The incidence rate is extremely high, which has seriously endangered human health. At present, it is considered that its pathogenesis is closely related to EB virus infection, chemical carcinogens, and genetic susceptibility genes [2, 3]. Radiotherapy is still the main treatment for NPC, but the local recurrence and distant metastasis easily occur after radiotherapy, which limits its ability to further improve the survival rate of patients [4]. The research on the related pathogenesis and metastasis mechanism of NPC is beneficial to the discovery of specific diagnostic indicators and gene therapy targets for NPC and has far-reaching significance.

Micro-RNAs (miRNAs) are a new class of highly conservative endogenous non-protein-encoding single-stranded small RNA molecules with a length of 21–30 nT, which have been discovered in recent years. It was accidentally discovered by Lee et al. in 1993 in *C. elegans*, with a length of about 22 nt, named lin-4-RNA. In 2000, Reinhart et al. found another important miRNA: let-7 posttranscriptional regulation: let-7 in wireworms. The discovery of lin-4 and let-7 kicked off the research on miRNA [5, 6]. With the improvement of research methods and the increasing attention paid to miRNA, more and more miRNA molecules are constantly revealed in a variety of organisms and become biomarkers for the diagnosis of diseases and tumors. Studies have shown that miR-338-3p becomes a tumor suppressor miRNA by inhibiting the proliferation, migration, and invasion of liver cancer, breast cancer, and ovarian cancer cells [7–9]. Research data have shown that the expression of miR-338-3p in gastric cancer is downregulated, and the degree of decrease is related to TNM staging. PTP1B may be a target gene of miR-338-3p, and the expression of PTP1B in gastric cancer may be regulated by miR-338-3p after transcription [10]. However, the relationship between miR-338-3p and NPC has not been studied systematically in depth.

Signal transduction and transcription activator 3(STAT3) is an oncogenic transcription factor commonly expressed in many tissues and plays an important role in regulating cell activity [11]. At the same time, it has a high expression level in many cancers and promotes tumorigenesis by preventing apoptosis, enhancing cell proliferation, and promoting angiogenesis, invasion, and metastasis [12–14]. Normally, the activation of STAT3 signals is tightly regulated and correlated with the degree of malignancy. In addition, STAT3 is a key transcriptional activation biomarker in tumor treatment, often associated with tumorigenesis. The latest research has shown that the invasion and migration of NPC cells are related to the activation of the STAT3 signaling pathway [15]. Therefore, we speculated that the detection of STAT3 expression in NPC may be an indicator of malignancy and prognosis and may provide a new target for tumor treatment. Therefore, this study mainly explored the expression changes of miR-338-3p in NPC tissues, as well as its relationship with STAT3 mRNA expression and the effects of both on clinical pathological parameters and prognosis of patients. The specific report is as follows.

## 2. Materials and Methods

### 2.1. Clinical Data

A total of 71 patients with NPC admitted to the Department of Otorhinolaryngology—Head and Neck Surgery—of Taizhou Hospital of Zhejiang Province affiliated to Wenzhou Medical University from February 2016 to February 2018 were selected as the nasopharyngeal carcinoma group. None of the patients received radiotherapy, chemotherapy, or other biological treatments, and was confirmed as primary NPC by postoperative pathological examination. A total of 71 cancer tissues were collected during the operation. There were 45 males and 26 females, and they were aged 40.32 ± 3.13 years old. Histological types: 43 cases with keratosis and 28 cases with nonkeratosis; clinical TNM staging included 30 cases in stages I-II and 41 cases in stages III-IV. Differentiation degree: 31 cases of medium and high differentiation squamous cell carcinoma and 40 cases of low undifferentiated carcinoma; there were 27 cases with distant metastasis and 44 cases without distant metastasis. Twenty-three patients who underwent biopsy due to chronic nasopharyngitis at the same period were selected as the control group, and 23 samples of nasopharyngeal mucosal tissue were collected. There were 14 males and 9 females aged 39.57 ± 3.26 years old. The gender and age of the two groups were comparable (*P* > 0.05). The study was reviewed by the hospital ethics committee, and informed consent forms were signed by the patients and their families.

### 2.2. Detection of miR-338-3p Expression in Nasopharyngeal Tissue

Two groups of nasopharyngeal tissues were selected. Total RNA was extracted with TRIzol reagent, and the concentration and purity of RNA were measured using an ultraviolet spectrophotometer. Tissue samples with good purity were selected for reverse transcription using a cDNA transcription kit (ThermoFisher). miR-338-3p primer sequence: forward: 5′-TGCGGTCCAGCATCAGTGAT-3′; reverse: 5′-CCAGTGCAGGGTCCGAGT-3′, U6 primer sequence: forward: 5′-TTCGGCAGCACATATAAATTGG-3′; reverse, 5′-CGCTTCAATTTGCGTGTCAT-3′, and considered as an internal reference. A reverse transcription reaction was performed in 50 ng of total RNA with a final volume of 10 *μ*L containing 0.1 pmol of specific primer, 1x reaction buffer, dNTP 10 nmol, and M-MLV RT 100 U. The reactants were incubated at 16 C for 30 min, 37 C for 50 min, and finally at 70 C for 15 min to terminate the reaction. Real-time fluorescent quantitative PCR amplification reaction was performed using a quantitative PCR instrument, with U6 as the internal reference. PCR reaction system: 1 *μ*L of RT product, 4 pmol of each primer, and 10 *μ*L of 2 × Evagreen Master Mix reagent. PCR reaction condition: 95°C, 30 s; 94°C, 10 s; and 61°C, 45 s, a total of 45 cycles. The 2^−ΔΔCt^ method [16] was used to calculate the relative expression level of miR-338-3p.

### 2.3. Determination of STAT3 Expression in Nasopharyngeal Tissue

Two groups of nasopharyngeal tissues were taken, and the total RNA was extracted and reversely transcribed into cDNA according to the method of reference 1.2. STAT3 primer sequence: forward: 5′-CGCACTTAGATTCATTGATGC-3′; reverse: 5′-AGGTGAGGACTCAAACTG-3′, GAPDH primer sequence: forward: 5′-TCAAGCAAGCAATGCC-3'; reverse: 5′-CGataCCAAAGTTGTCATGGA-3′, which was considered as the internal reference. The reactants were incubated at 16°C for 30 min, 37°C for 50 min, and finally at 70°C for 15 min to terminate the reaction. Real-time fluorescent quantitative PCR amplification reaction was performed using a quantitative PCR instrument, with GAPDH as the internal reference. PCR reaction system: 1 *μ*L of RT product, 4 pmol of each primer, and 10 *μ*L of 2 × Evagreen Master Mix reagent. PCR reaction condition: 95°C, 30 s; 95°C, 5 s; 60°C, 33 s, a total of 40 cycles. The 2^−ΔΔCt^ method [16] was used to calculate the relative expression of STAT3.

### 2.4. Follow-Up

All patients received surgical treatment, and they were followed up by telephone, outpatient, and other means after discharge, about once a month. The follow-up period ended in February 2021.

### 2.5. Statistical Methods

SPSS 19.0 statistical software was used for analysis of the data, and the gender, age, histological type, clinical TNM stage, T stage, N stage, M stage, and differentiation degree of NPC patients were recorded. Measurement data were expressed as mean ± standard deviation, and measurement data subject to normal distribution were compared between two groups using *t*-test and paired *t*-test. Count data were expressed as percentage and rate using Chi-square test. *P* < 0.05 indicated that the difference was statistically significant. The Pearson correlation analysis was used to analyze the correlation between miR-338-3p and STAT3, and the Kaplan–Meier method was used to compare the two with the survival rate.

## 3. Results

### 3.1. Comparison of miR-338-3p and STAT3 mRNA Expression in Nasopharyngeal Tissue between the Two Groups

The results showed that the relative expression levels of miR-338-3p in nasopharyngeal tissues of the NPC group and the control group were 0.39 ± 0.05 and 1.01 ± 0.09, respectively. The relative expression levels of STAT3 mRNA in nasopharyngeal tissues of the NPC group and the control group were 3.82 ± 0.21 and 1.04 ± 0.11 respectively. Compared with the control group, the mRNA expression of miR-338-3P was downregulated and the mRNA expression of STAT3 was upregulated in the nasopharyngeal carcinoma group (both *P* < 0.05, Figures 1(a) and 1(b)).

### 3.2. Analysis of Correlation between miR-338-3p and STAT3

Pearson correlation analysis showed a statistically significant weak negative correlation between miR-338-3p and STAT3 (*r* = −0.523, *P* < 0.001, Figure 2).

### 3.3. Comparison of miR-338-3p Expression in NPC Tissues between Different Clinical Pathological Parameters in Patients with NPC

The comparison of the expression of miR-338-3p in NPC tissues among different clinical pathological parameters in patients with NPC showed that the low expression of miR-338-3p was related to the age (<30) of the patient, clinical TNM stage (III∼IV), T stage (*T*_3_∼*T*_4_), and distant metastasis (yes) (all *P* < 0.05, Table 1).

### 3.4. Comparison of STAT3 Expression in NPC Tissues between Different Clinical Pathological Parameters in Patients with NPC

The comparison of STAT3 expression in NPC tissues among different clinical pathological parameters in NPC patients revealed that the high expression of STAT3 was related to the clinical TNM stage (III∼IV), T stage (*T*_3_∼*T*_4_), and distant metastasis (Yes) in these patients (all *P* < 0.05, Table 2).

### 3.5. miR-338-3p Expression and Prognosis of NPC Patients

A total of 71 NPC patients were followed up for three years. By February 2021, three patients were lost to follow-up and 13 patients died. With the mean of miR-338-3p 0.39 as the boundary, they were divided into a miR-338-3p low expression group (*n* = 36) and a miR-338-3p high expression group (*n* = 32). The survival rate of the miR-338-3p low-expression group was 69.44%, which was lower than that of the miR-338-3p high-expression group (93.75%). The difference was statistically significant (log-rank = 6.436, *P* = 0.011, Figure 3).

### 3.6. Relationship between STAT3 Expression and Prognosis of NPC

There were 71 patients with nasopharyngeal carcinoma, 3 cases lost to follow-up and 13 cases died. Defined by the mean of STAT3 (3.82), they were divided into a STAT3 low-expression group (37 cases) and a STAT3 high-expression group (31 cases). The survival rate of the STAT3 high-expression group was 67.57%, while that of the STAT3 low-expression group was 96.77%, and the difference was statistically significant (log-rank = 5.743, *P* = 0.017, Figure 4).

## 4. Discussion

NPC is a secretive disease with no obvious clinical manifestation in the early stage, which is not easy to be detected, and the lymph node metastasis of NPC occurs early. Therefore, early diagnosis of NPC is particularly important in China. At present, the clinical screening for NPC is mainly to detect the EB virus infection in the blood, such as EBv-DNA and EBV-VCA-IgA. However, NPC is not completely related to EBV, and many diseases (such as lymphoma, gastric cancer, breast cancer, pharyngitis, and infectious mononucleosis) can be accompanied by EBV infection. A certain proportion of healthy people are infected [17]. A large number of clinical practices have proved that the sensitivity and specificity of EBV-related detection in the diagnosis of NPC are not high, which cannot meet the requirements of being used as an early diagnostic marker [18]. A good molecular marker screening method should be minimally invasive and repeatable, and ideally tumor tissue-specific molecules can be detected with a simple blood or urine test. In addition, screening techniques should be sensitive enough to detect early stage cancer while accurately differentiating individuals without cancer. Finding ideal molecular markers and methods for early diagnosis and monitoring of NPC is an urgent problem to be solved in the prevention and treatment of NPC.

With the improvement of research methods and the increasing attention paid to miRNA, more and more miRNA molecules are revealed in diseases [19]. miRNAs exert regulatory effects mainly by inhibiting their target genes. One mode of action is incomplete complementary binding to the 3′ untranslated region (UTR) of the target gene, thereby inhibiting translation without affecting the stability of miRNA. The other one is completely and complementarily combined with the target gene 3′UTR, with the action mode and function very similar to that of siRNA, finally leading to the degradation of target mRNA. Recently, a third mode has also been found, that is, miRNAs direct the rapid deadenylation of mRNA of their target genes, resulting in rapid mRNA attenuation and decreased expression levels. Studies have shown that the downregulation of miR-338-3p is associated with worse cell differentiation and later lymph node staging in NSCLC [20], suggesting that miR-338-3p may be involved in the growth and metastasis of primary tumors.

However, the specific regulatory mechanisms may vary among tissues of different tumors. In our study, we also found that the expression of miR-338-3p was downregulated and indicated that the underexpression of miR-338-3p might be related to the development of NPC patients. In this study, we analyzed the relationship between the expression of miR-338-3p in NPC tissue and clinical pathological parameters of patients. It was found that the expression of miR-338-3p in NPC tissue in patients younger than 30 years old (young type) was lower than that in patients ≥3 years old, suggesting that young patients may have unique carcinogenic pathways and clinical and biological characteristics. Previous studies have shown that young patients with NPC have less expression of p53 and Bcl-2, two key proteins that control the balance of apoptotic survival, and less IgA anti-EA and anti-VCA antibodies [21], and more C-kit receptors and EBV-related cancer protein LMP1 [22]. This may be one of the reasons for the decrease of miR-338-3p in young NPC patients, but the specific mechanism needs further investigation. The results of this study also showed that the expression of miR-338-3p in the NPC tissue with lymph node and/or distant metastasis, clinical TNM stage III-IV, and T stage T3-T4 were lower than those in the NPC tissue without metastasis, clinical TNM stage I-II, and T stage *T*1∼*T*2. This indicates that the low expression of miR-338-3p may participate in the proliferation, migration, and invasion of cancer cells.

STAT, a family of proteins with special significance in cells, is encoded by the STAT gene and is an important transcription factor in the process of cell proliferation, maturation, and survival. It can affect the proliferation of tumor cells and normal cells, help promote the metastasis and differentiation of tumor cells, and inhibit the apoptosis of tumor cells [23]. Among them, STAT3 is most closely related to cancer, and its abnormal activation is closely related to the occurrence and development of a variety of human malignant tumors, such as leukemia, lymphoma, prostate cancer, and all kinds of head and neck tumors and gastrointestinal tumors as well as to immune tolerance in the tumor microenvironment [24]. Studies have shown that the expression level of STAT3 protein in NPC tissue is significantly higher than that in normal nasopharyngeal tissue, and its expression is positively correlated with clinical staging [25], indicating that the expression of STAT3 and STAT 3 is closely related to the occurrence and development of NPC and provides a theoretical basis for searching molecular markers of NPC. In this study, we detected STAT3 expression levels in NPC tissues from patients with NPC and nasal mucosa tissues from patients with nasopharyngitis, and the results confirmed an upregulation of STAT3 in gastric carcinoma, which is consistent with STAT3 expression in the TCGA database. Bioinformatics analysis indicated that STAT3 might be a downstream target gene of miR-338-3p. Correlation analysis showed that miR-338-3p was negatively correlated with STAT3, indicating that miR-338-3p might negatively regulate STAT3 expression. Analysis of the relationship between STAT3 expression in NPC and clinical pathological parameters showed that STAT3 was also related to clinical TNM stage, T stage, and distant metastasis in patients, suggesting that STAT3 was also involved in the proliferation and diffusion of cancer cells.

Analysis of the relationship between miR-338-3p, STAT3, and the prognosis of NPC patients revealed that the survival rate in the miR-338-3p low expression group was significantly lower than that in the miR-338-3p high expression group. The survival rate of patients in the STAT3 high expression group was significantly lower than that of the STAT3 low expression group, suggesting that miR-338-3p is low expressed in NPC patients, and patients with high expression of STAT3 should focus on monitoring the development of the disease to prevent its deterioration.

## 5. Conclusion

To sum up, low expression of miR-338-3p and high expression of STAT3 in NPC patients are related to the clinical features and prognosis of the patients. However, whether miR-338-3p and STAT3 can be used as molecular markers for detecting the condition of NPC patients needs to be further explored by expanding the sample size, and the effects of the two on the biological behavior of cancer cells can be explored in subsequent studies, so as to provide more new reference basis for molecular targeted therapy for NPC.

## Figures and Tables

**Figure 1:** Comparison of miR-338-3p and STAT3 mRNA expression in nasopharyngeal tissues between the two groups. *Note.* Compared with the control group, ^*∗*^*P* < 0.05.

**Figure 2:** Correlation analysis between miR-338-3p and STAT3.

**Figure 3:** The relationship between the expression of miR-338-3p and the prognosis of patients with nasopharyngeal carcinoma.

**Figure 4:** The relationship between the expression of STAT3 and the prognosis of patients with nasopharyngeal carcinoma.

**Table 1:** Comparison of miR-338-3p expression in nasopharyngeal carcinoma tissues among different clinicopathological parameters of nasopharyngeal carcinoma patients.

Pathological parameters	*n*	miR-338-3p	T value	*P* value
Gender				
Male	45	0.37 ± 0.04	1.684	0.097
Female	26	0.39 ± 0.06		
Age (years)				
≥30	62	0.42 ± 0.05	2.716	0.025
<30	9	0.38 ± 0.04		
Histological type				
Nonkeratinized	28	0.37 ± 0.05	0.731	0.467
Keratinized	43	0.38 ± 0.06		
Clinical TNM staging				
I∼II	30	0.44 ± 0.07	5.817	<0.001
III∼IV	41	0.35 ± 0.06		
T staging				
T_1_∼T_2_	22	0.42 ± 0.06	2.903	0.005
T_3_∼T_4_	49	0.37 ± 0.07		
N staging				
N_1_∼N_2_	18	0.40 ± 0.06	0.611	0.543
N_3_∼N_4_	53	0.41 ± 0.07		
M staging				
M_0_	61	0.38 ± 0.07	0.877	0.384
M_1_	10	0.36 ± 0.04		
Differentiation				
Medium and high differentiation	31	0.40 ± 0.04	1.820	0.073
Low, undifferentiated	40	0.38 ± 0.05		
Distant metastasis				
No	44	0.41 ± 0.07	3.236	0.002
Yes	27	0.36 ± 0.05		

**Table 2:** Comparison of STAT3 expression in nasopharyngeal carcinoma tissues among different clinicopathological parameters of nasopharyngeal carcinoma patients.

Pathological parameters	*n*	miR-338-3p	T value	*P* value
Gender				
Male	45	3.81 ± 0.18	0.433	0.666
Female	26	3.79 ± 0.20		
Age (years)				
≥30	62	3.76 ± 0.21	1.056	0.295
<30	9	3.84 ± 0.23		
Histological type				
Nonkeratinized	28	3.83 ± 0.18	0.214	0.831
Keratinized	43	3.84 ± 0.20		
Clinical TNM staging				
I∼II	30	3.74 ± 0.16	5.184	<0.001
III∼IV	41	4.01 ± 0.25		
T staging				
T_1_∼T_2_	22	3.80 ± 0.19	3.030	0.003
T_3_∼T_4_	49	3.97 ± 0.23		
N staging				
N_1_∼N_2_	18	3.79 ± 0.17	0.730	0.468
N_3_∼N_4_	53	3.83 ± 0.21		
M staging				
M_0_	61	3.81 ± 0.22	0.406	0.686
M_1_	10	3.84 ± 0.19		
Differentiation				
Medium and high differentiation	31	3.78 ± 0.18	1.745	0.085
Low, undifferentiated	40	3.86 ± 0.20		
Distant metastasis				
No	44	3.75 ± 0.23	2.464	0.016
Yes	27	3.88 ± 0.19		

## Data Availability

The data used and analyzed during the current study are available from the corresponding author on reasonable request.
